This article has been retracted.

# Breast Cancer Classification Prediction Based on Ultrasonic Image Feature Recognition

**DOI:** 10.1155/2021/4025597

**Published:** 2021-09-24

**Authors:** Yihong Huang, Shuo Zheng, Yu Lin, Haiyan Miao

**Affiliations:** ^1^Department of Ultrasound Diagnosis, Fuzhou Second Hospital Affiliated to Xiamen University, Fuzhou 350007, China; ^2^Department of Hepatobiliary Surgery, Fuzhou Second Hospital Affiliated to Xiamen University, Fuzhou 350007, China; ^3^Department of General Surgery, The Sixth People's Hospital of Nantong, Nantong, Jiangsu 226001, China

## Abstract

Exploring an effective method to manage the complex breast cancer clinical information and selecting a suitable classifier for predictive modeling still require continuous research and verification in the actual clinical environment. This paper combines the ultrasound image feature algorithm to construct a breast cancer classification model. Furthermore, it combines the motion process of the ultrasound probe to accurately connect the ultrasound probe to the breast tumor. Moreover, this paper constructs a hardware and software system structure through machine vision algorithms and intelligent motion algorithms. Furthermore, it combines coordinate transformation and image recognition algorithms to expand the recognition process to realize automatic and intelligent real-time breast cancer diagnosis. In addition, this paper combines machine learning algorithms to process data and obtain an intelligent system model. Finally, this paper designs experiments to verify the intelligent system of this paper. Through experimental research, it can be seen that the breast cancer classification prediction system based on ultrasonic image feature recognition has certain effects.

## 1. Introduction

Breast cancer is one of the high-incidence diseases in women, and its morbidity and mortality account for the first place in female malignant tumors [1]. Therefore, accurate diagnosis of breast cancer is of great significance for subsequent treatment. Among them, histopathological diagnosis is regarded as the “gold standard” for tumor diagnosis. There is a potential relationship between the cell structure and spatial distribution in the tissue. The diseased tissue is different from normal tissue in terms of morphology and cell spatial distribution [2]. Factors such as morphological changes, neighboring relationships, and spatial distribution between tissue structures also play an important role in disease diagnosis. Moreover, pathologists use time-consuming and laborious diagnoses in clinical diagnosis by observing the morphology and distribution of cells, and the diagnosis results are easily affected by subjective factors such as the pathologist's experience and knowledge level. Therefore, it is necessary to use computer-aided diagnosis to analyze and diagnose pathological images, providing doctors with more objective and reliable diagnosis results [3].

Breast cancer will produce a series of mutations in the continuous division of tumor cells and produce some unknown biochemical reactions, resulting in different biological characteristics from normal cells. Therefore, due to the individual specificity of different patients, there will be different changes, and their course of disease development, treatment effect, metastasis status, and recurrence probability are not the same. The above characteristics also determine that the diagnosis basis of breast cancer has multiple sources of relevance, the high sequence relevance of the diagnosis and treatment process, and the diversity of postoperative recurrence factors. Accurate diagnosis of breast cancer involves many data, wide dimensions, and strong physical and chemical indicators heterogeneity. Due to the limited medical resources and the further pursuit of improving the accuracy of diagnosis and treatment, machine learning can help doctors greatly improve their work efficiency in breast cancer classification, diagnosis, and prognosis. The consideration dimensions include the choice of examination methods and the diagnosis of breast cancer types, according to the patient's medical history, physical state, psychology, the affordable economic conditions of the patient's home, the potential for postoperative recurrence and metastasis, and treatment response prediction and treatment. Each dimension involves multiple subdimensions and a large amount of data analysis. The inspection method alone includes biochemical inspection, imaging inspection, pathological biopsy, and other methods. Each inspection corresponds to a large number of physical and chemical indicators. In addition, these physical and chemical indicators are also heterogeneous. It is common to have different breast cancers, but the physical and chemical indicators are very similar, or the same type of breast cancer has different pathological characteristics. These factors often bring huge challenges to the accurate diagnosis, precise treatment, and postoperative breast cancer follow-up. In the actual clinical diagnosis of breast cancer, the patient will be asked to perform some cost-effective and routine examinations, such as blood tests and mammography, for preliminary screening; second, the doctor will decide to conduct more precise special examinations, such as blood tumor markers, based on the patient's condition, examination, breast CT, and so on; and finally, according to the preliminary examination, if the condition requires more precise traumatic examinations such as fine/thick needle aspiration biopsy of the breast, immunohistochemistry will be performed. Different types of clinical examinations have different data characteristics, different evaluation criteria, and different levels of importance of different indicators. Therefore, when using artificial intelligence methods to assist breast cancer diagnosis, different examinations are suitable for different models. Whether these data with different characteristics should be treated independently or as a complete problem to model is a key. From the clinical medicine perspective, effective breast cancer diagnosis must be derived from multisource data. Multifactor features are used as input. There are more combination possibilities between features and classifiers, such as whether a factor feature should be input into a classifier, or all features should be input as a single feature into a classifier. This further increases the modeling complexity of the problem because different classifiers may classify different information, and people expect to obtain a more reliable model by maximizing the use of this information, rather than choosing the best one from the available classifiers. The decision-making process is further complicated by the absence of established assessment methods for classifier performance, such as repeatability and clinical practicability.

## 2. Related Work

Literature [4] used feature descriptors such as local binary patterns, gray-level cooccurrence matrices, and classification models such as random forests and support vector machines to achieve a recognition rate of about 85% on medical data sets. Literature [5] used local binary patterns of opposite colors, Gabor features, and other descriptors and classification models such as support vector machines and decision trees. Moreover, it integrated the results of each classification model through the majority voting strategy and achieved a recognition rate of 87% on the same data set. Feature descriptors are difficult to describe completely different pathological images and are sensitive to scale and morphological changes. The extraction of high-quality features requires corresponding professional knowledge and energy, limiting the application of this method. The classification algorithm based on deep learning uses the network structure with the convolutional layer as the core to achieve a more effective feature learning process, so it has better performance than traditional machine learning classification algorithms. Literature [6] applied deep learning to breast cancer pathological images, used 11-layer and 13-layer deep neural networks to classify mitosis in the input image, and applied the classification results to subsequent mitosis detection tasks. Literature [7] used a 14-layer convolutional neural network to classify breast pathological images into normal tissues/benign lesions/carcinoma in situ. Literature [8] used a model based on AlexNet to perform experiments, which has achieved a performance improvement of 4% to 6% compared with machine learning classification algorithms. Literature [9] used a deep network based on independent magnification to achieve a recognition rate of 83% on the same data set. Literature [10] used a classification model based on Fisher vectors and VGGNet to achieve a recognition rate of 87%. Although deep networks can better complete the task of classification of breast cancer pathological images, there are some problems. For example, there are great differences between pathological images under different magnifications, and maintaining good robustness to pathological images under different magnifications is the key to the task. In addition, deep network training requires many training samples, and the number of breast cancer pathological images available for research is limited. Making good use of the limited samples is the key to improving the performance of the classification model [11]. The channel recalibration model is an attention model that acts on the feature channel domain. The channel weights learned in the training process are used to suppress useless features and improve the performance of the classification model. In order to make better use of the feature information in the convolutional neural network, literature [12] proposed a multiscale channel recalibration model based on the channel recalibration model, using different maximum pooling layers to obtain multiscale features.

Moreover, it performed channel recalibration for each scale feature separately. It merged the channel weights as the final channel weight, thereby achieving multiscale channel recalibration for input features. Multiscale features can enrich the feature information in the network, and the channel recalibration model combined with multiscale features can further improve the performance of the classification model. In addition, the training set of the network is composed of pathological images of breast cancer under four magnifications, which can ensure that the classification model is robust to pathological images under different magnifications to better meet clinical needs [13].

Literature [14] studied tumor genes, selected tumor gene expression profiles as key sample data, and used a combination of SVM and PCA to identify the types of colon cancer. The results of the experiment show that the accuracy of the model can reach 95.16%. Literature [15] normalized the logistic equation into linear regression to deal with logistic regression classification. This kind of normalization can effectively suppress background noise and have good rationality to ensure that the model's main focus is on the key feature data to facilitate the extraction of rules. Finally, literature [16] used the genetic algorithm to randomly extract features in a machine learning model and then merged multiple networks to form the final model.

## 3. Ultrasound Image Recognition Algorithm

The reference coordinate system of the ultrasonic recognition image system is the mechanical coordinate system of the ultrasonic probe and each subdevice. For example, the mechanical coordinate system of the ultrasonic probe system shown in Figure 1 is defined as follows [17].

The origin *O* in Figure 1 is the geometric center of the end face of the ultrasound probe system and the breast tumor. The *X*-axis is along the longitudinal axis of the ultrasonic probe one by one, and the ultrasonic probe motion orbiter points to the direction of the ultrasonic probe rising mechanism. The *Z*-axis is located in the butt surface of the ultrasound probe system and the breast tumor one by one and is perpendicular to the *X*-axis. The *Y*-axis is determined according to the *XZ*-axis in the right-hand system.

(1) The mechanical coordinate system of the ultrasonic probe motion orbiter is OG-XGYGZG. The *OG*-axis runs along the longitudinal axis of the ultrasound probe, the *XG*-axis runs along the longitudinal axis of the ultrasound probe, the *ZG*-axis runs along the docking surface of the ultrasound probe system and the breast tumor, and the *YG*-axis follows the *ZG* and *XG* axes of the right-hand system [18].

(2) The ascending mechanism of the ultrasonic probe's mechanical coordinate system is OP-XPYPZP. The *XP*-axis is perpendicular to the bottom surface of the ultrasonic probe raising mechanism and points in the direction of the passive component of the rendezvous and docking mechanism, and the origin OP is located at the geometric center of the connecting surface between the lower plane of the ultrasonic probe raising mechanism and the ultrasonic probe raising mechanism. The *ZP*-axis is perpendicular to the *XP*-axis, perpendicular to the measurement and control antenna mounting surface, and the pointing rendezvous is positive for the approaching field's target marker.

The ultrasonic probe motion orbiter's mechanical coordinate system is identical to the ultrasonic probe's mechanical coordinate system, and the +*Z*-axis points to the I quadrant line. From its rear end surface, the ultrasonic probe motion orbiter faces forward (pointing to the ultrasonic probe motion orbiter's support cabin structure) along the longitudinal axis (the longitudinal geometric axis of the ultrasonic probe motion orbiter's housing). In addition, the clockwise quadrants are renamed I, II, III, and IV, and the quadrants are divided by 90°.

The mechanical coordinate system of the returner's coordinate origin is situated at the center circle point of the returner's back-end frame. Therefore, the origin of the coordinate system has been changed.

The status of the combination is shown in Figure 2.

(3) The docking mechanical coordinate system of the orbit-back assembly is OGD-XGDYGDZGD. The origin OGD is located at the geometric center of the mechanical installation surface of the active part of the ultrasonic probe motion orbiter docking mechanism and the ultrasonic probe motion orbiter. The *XGD*-axis is perpendicular to the mechanical mounting surface of the active part of the docking mechanism and the ultrasonic probe motion orbiter and points to the same direction as the *XGD*-axis of the mechanical coordinate system of the ultrasonic probe motion orbiter. The *ZGD*-axis is perpendicular to the *XGD*-axis, and its pointing is the same as the *ZG*-axis of the mechanical coordinate system of the ultrasonic probe motion orbiter. When the rendezvous and docking are oriented toward the moon, the *ZGD* axis points to the moon, as shown in Figure 3. The *YGD*-axis and the *ZGD* and *XGD* axes constitute a right-handed rectangular coordinate system [19].

(4) The docking mechanical coordinate system of the ultrasonic probe rising mechanism is OPD-XPDYPDZPD. The origin OPD is located at the geometric center of the mechanical installation surface of the passive component of the ultrasonic probe rising mechanism docking mechanism and the ultrasonic probe rising mechanism. The *XPD*-axis is perpendicular to the mechanical mounting surface of the passive part of the docking mechanism and the ultrasonic probe rising mechanism and points to the passive part of the ultrasonic probe rising mechanism butting mechanism. The *ZPD*-axis is perpendicular to the *XPD*-axis, and the direction is the same as the *ZP*-axis of the mechanical coordinate system of the ultrasonic probe ascending mechanism.

The coordinate system of a machine vision system generally includes the following three coordinate systems: world coordinate system, camera coordinate system, and image coordinate system. The following coordinate systems are established in the OpenCV standard, which can be transformed between the corresponding coordinate systems.

1. The world coordinate system: generally speaking, the world coordinate system can be established on a certain point of the target object. In this way, since the size information of the characteristic points in the target object is known, it can be obtained that each characteristic point is in the world coordinate system. In the coordinates, generally, the geometric center of the target object can be selected as this point. In this paper, the geometric center of the plane of the ultrasonic probe rising mechanism and the ultrasonic probe motion orbiter is selected as the origin. The role of the world coordinate system can be summarized in two points: first, the geometric relationship of the feature points is transformed into its coordinates in the world coordinate system after its establishment; and second, the world coordinate system provides a camera that has nothing to do with the camera's imaging process.
2. Camera coordinate system: the optical center of the camera lens is the origin of the camera coordinate system. Generally, the *X* and *Y* axes of the image coordinate system are pointed to as the *X* and *Y* axes of the camera coordinate system. The *Z*-axis can be determined according to the *XY-*axis coordinates and the right-hand system.
3. Image coordinate system: the image coordinate system, as its name implies, is a coordinate system established on the image. Unlike the other two coordinate systems, it is a coordinate system on a plane with only the *XY*-axis. The origin of the image coordinate system is the center of the image plane, that is, the projection of the main optical axis of the camera on the plane. The *XY*-axis of the pixel coordinate is set to the *XY*-axis direction of the image coordinate system.

The relationship between the three coordinate systems is shown in Figure 4 [20].

As shown in Figure 4, OCXCYCZC is the camera coordinate system, in which OCZC is the main optical axis direction, OXY is the image coordinate system, О is the projection of the main optical axis on the imaging plane, and OWXWYWZW is the world coordinate system.

The pixel coordinates and the coordinates in the image coordinate system are in a translational relationship, as shown in Figure 5.

The OUV rectangular coordinate system is defined in Figure 5, the pixel point (*u*, *v*) represents the number of rows and columns of the pixel, and the pixel is the unit in the coordinate system. Thus, an image coordinate system with the physical length as the coordinate system and the image center as the origin Oc is established. The *XY*-axis is parallel to the UV-axis, respectively. In the original coordinate system, Oc coordinates (*u*0, *v*0), the coordinate offset of a pixel is d*x*, and d*y* (on the *XY*-axis) is the pixel size [21]:

(1) $$\begin{array}{c} \left\{\begin{array}{c} u=\frac{x}{dx}+u_{0},\\ v=\frac{y}{dy}+v_{0}. \end{array}\right. \end{array}$$

The world coordinate system and the camera coordinate system, respectively, correspond to the ultrasonic probe ascending mechanism coordinate system and the translated ultrasonic probe motion orbiter coordinate system. Their relative pose relationship is the relative pose of the camera and the target object. For point Р, its coordinates in the world coordinate system are (XW, YW, ZW), and the coordinates in the camera coordinate system are (XC, YC, ZC). The relationship between them is as follows:

(2) $$\begin{array}{c} \left[\begin{array}{c} X_{c}\\ y_{c}\\ z_{c} \end{array}\right]=R\left[\begin{array}{c} X_{W}\\ y_{W}\\ z_{W} \end{array}\right]+t. \end{array}$$

Among them, *R* is the three-dimensional rotation matrix, which is an orthogonal matrix, *t* is the translation vector, and the relationship is as follows:

(3) $$\begin{array}{c} R=\left[\begin{array}{ccc} r_{11} & r_{12} & r_{13}\\ r_{21} & r_{22} & r_{23}\\ r_{31} & r_{32} & r_{33} \end{array}\right]\;t=\left[\begin{array}{c} t_{x}\\ t_{y}\\ t_{z} \end{array}\right]. \end{array}$$

For this subject, the ultimate goal is to calculate the rotation matrix *R* and the translation vector *t*.

In the ultrasonic probe vision measurement system, the dual-spectrum camera is the perspective imaging model and the pinhole imaging model. Therefore, it is an ideal perspective projection imaging model and ignores the distortion of the camera, as shown in Figure 6.

As shown in Figure 6, the length of ocol is the focal length *f*. According to the principle of similar triangles, it is easy to get the following formula [22]:

(4) $$\begin{array}{c} \left\{\begin{array}{c} x=\frac{fX_{c}}{Z_{c}},\\ y=\frac{fY_{c}}{Z_{c}}. \end{array}\right. \end{array}$$

Among them, (*x*, *y*) are the coordinates of point *p* in the image coordinate system and (*XC*, *YC*, *ZC*) are the coordinates in the camera coordinate system. The perspective projection relationship can be expressed as a matrix as follows:

(5) $$\begin{array}{c} Z_{c}\left[\begin{array}{c} x\\ y\\ 1 \end{array}\right]=\left[\begin{array}{cccc} f & 0 & 0 & 0\\ 0 & f & 0 & 0\\ 0 & 0 & 1 & 0 \end{array}\right]\left[\begin{array}{c} X_{c}\\ Y_{c}\\ Z_{c}\\ 1 \end{array}\right]. \end{array}$$

From the above equations, the following relationship (6) can be obtained. The camera's internal parameters determine the matrix M1, and the position matrix of the physical coordinate system and the camera coordinate system is M2. The internal parameters of the camera need to be calibrated in advance, so M1 is known. It can be concluded from the theory of visual projection imaging that when the coordinates of a certain number of points in the world coordinate system and the corresponding image plane coordinates are known, the pose matrix in the following formula can be obtained:

(6) $$\begin{array}{c} Z_{c}\left[\begin{array}{c} u\\ v\\ 1 \end{array}\right]=\left[\begin{array}{ccc} \frac{1}{dx} & 0 & u_{0}\\ 0 & \frac{1}{dy} & v_{0}\\ 0 & 0 & 1 \end{array}\right]\left[\begin{array}{cccc} f & 0 & 0 & 0\\ 0 & f & 0 & 0\\ 0 & 0 & 1 & 0 \end{array}\right]\left[\begin{array}{cc} R & t\\ 0 & 1 \end{array}\right]\left[\begin{array}{c} X_{W}\\ Y_{W}\\ Z_{W}\\ 1 \end{array}\right]=M_{1}M_{2}\left[\begin{array}{c} X_{W}\\ Y_{W}\\ Z_{W}\\ 1 \end{array}\right]=M\left[\begin{array}{c} X_{W}\\ Y_{W}\\ Z_{W}\\ 1 \end{array}\right]. \end{array}$$

*M* is called the projection matrix, which describes the one-to-one correspondence between the image points in the image and the feature points of the target object. According to the analysis of the above formula, the measurement problem in this paper can be abstracted as follows.

The target feature point is a set of object point coordinates P (XW, YW, ZW) in the world coordinate system, the corresponding image point coordinates P′(*u*, *v*) and internal parameters such as the focal length of the camera are set. Moreover, it is necessary to solve for ZC and the rotation matrix *R* and the translation matrix T. According to these two matrices, the relative pose of the ultrasound probe is obtained.

How to describe the rotation of a rigid body in three-dimensional space is an interesting problem. In the PnP problem, a rotation matrix is used to describe the rotation of a rigid body, but the relationship between the rotation angle and the rotation matrix is worth studying.

### 3.1. Rotation Matrix

The matrices that rotate around the *X*-axis, *Y*-axis, and *Z*-axis are formulas (7), (8), and (9), respectively:

(7) $$\begin{array}{c} R_{x}\left(\psi \right)=\left[\begin{array}{ccc} 1 & 0 & 0\\ 0 & \cos\;\psi & -\sin\;\psi \\ 0 & \sin\;\psi & \cos\;\psi \end{array}\right], \end{array}$$

(8) $$\begin{array}{c} R_{x}\left(\theta \right)=\left[\begin{array}{ccc} \cos\;\theta & 0 & \sin\;\theta \\ 0 & 1 & 0\\ -\sin\;\theta & 0 & \cos\;\theta \end{array}\right], \end{array}$$

(9) $$\begin{array}{c} R_{z}\left(\phi \right)=\left[\begin{array}{ccc} \cos\;\phi & -\sin\;\phi & 0\\ \sin\;\phi & \cos\;\phi & 0\\ 0 & 0 & 1 \end{array}\right]. \end{array}$$

Obviously, any rotation in any three-dimensional space can be decomposed into a certain angle around the *X*, *Y*, and *Z* axes. Euler angles describe rotation in this way.

### 3.2. Euler Angle

Euler angles are used to describe rotation in three-dimensional space. The rotation matrix can be seen as a combination of three rotations around the *X*, *Y*, and *X* axes. Because matrix multiplication does not satisfy the commutative law, different rotation orders will affect the final result, so a fixed order is required to accurately describe a rotation. This article stipulates that all rotations are rotated around the *X*-axis, *Y*-axis, and *Z*-axis in turn, and the resulting rotation matrix is shown in the following formula:

(10) $$\begin{array}{c} R=R_{Z}\left(\phi \right)R_{y}\left(\theta \right)R_{x}\left(\psi \right)\\ =\left[\begin{array}{ccc} \cos\;\theta \;\cos\;\phi & \sin\;\psi \;\sin\;\theta \;\cos\;\phi -\cos\;\psi \;\sin\;\phi & \cos\;\psi \;\sin\;\theta \;\cos\;\phi +\sin\;\psi \;\sin\;\phi \\ \cos\;\theta \;\sin\;\phi & \sin\;\psi \;\sin\;\theta \;\sin\;\phi +\cos\;\psi \;\cos\;\phi & \cos\;\psi \;\sin\;\theta \;\sin\;\phi -\sin\;\psi \;\cos\;\phi \\ -\sin\;\theta & \sin\;\psi \;\cos\;\theta & \cos\;\psi \;\cos\;\theta \end{array}\right]. \end{array}$$

It can be known from formula (10) that the rotation matrix can be obtained by knowing three Euler angles. Correspondingly, when a rotation matrix *R* is known, the Euler angle can also be calculated:

(11) $$\begin{array}{c} \psi =a\;\tan\;2\left(R_{32},R_{33}\right), \end{array}$$

(12) $$\begin{array}{c} \theta =a\;\tan\;2\left(-R_{31},\sqrt{R_{32}^{2}+R_{33}^{2}}\right), \end{array}$$

(13) $$\begin{array}{c} \phi =a\;\tan\;2\left(R_{21},R_{11}\right). \end{array}$$

The rotation matrix *R* can compute three rotation angles using formulas (11)–(13). The position and posture of the ultrasonic probe rising mechanism in the ultrasonic probe moving orbiter coordinate system are computed using the position and posture of the ultrasonic probe moving orbiter and the ultrasonic probe rising mechanism in the space coordinate system.

The relationship between coordinate systems A and B (both A and B have no offset): when A rotates 90° around the *Y*-axis and then rotates 90° around the *Z*-axis, we get B (counterclockwise is positive). If RABPA = PB, PA, and PB are a set of coordinate matrices of points in coordinate systems A and B, then

(14) $$\begin{array}{c} R_{\mathrm{AB}}=R_{Z}\left(\phi \right)R_{y}\left(\theta \right)=\left[\begin{array}{ccc} 0 & -1 & 0\\ 1 & 0 & 0\\ 0 & 0 & 1 \end{array}\right]\left[\begin{array}{ccc} 0 & 0 & 1\\ 0 & 1 & 0\\ -1 & 0 & 0 \end{array}\right]=\left[\begin{array}{ccc} 0 & -1 & 0\\ 0 & 0 & 1\\ -1 & 0 & 0 \end{array}\right]. \end{array}$$

Suppose we want to know the deviation between the actual coordinate system and the standard coordinate system. In that case, we need to multiply the result *R* and the inverse of RAB, so that the rotation matrix obtained is the deviation between the standard and the actual.

## 4. Evaluation of the Prediction Effect of Breast Classification Based on Ultrasound Image Features

The breast cancer detection classification model based on ultrasonic image feature recognition proposed in this study is shown in Figure 7. The model's overall structure is divided into two modules: lesion location module and lesion fine classification module. The lesion location module is used to detect suspected areas, reduce false negatives, and improve sensitivity. The lesion fine classification module is used to further classify and identify the suspected area and determine whether the suspected area is a lesion.

Image analysis mainly uses digital image processing technology to extract useful information from images, including image preprocessing, texture analysis, and feature dimensionality reduction, which correspond to different stages of image processing in turn. The image analysis process is shown in Figure 8.

After building a breast cancer detection classification model based on ultrasound picture feature identification, the model is tested, validated, and evaluated. Multiple sets of data are used to assess the system's performance, and a significant number of ultrasound pictures are gathered through the network to create a test database.

The impact of the system developed in this article is validated, and the accuracy of breast cancer detection and classification based on ultrasonic image feature identification is tallied after acquiring the database.

The results obtained are shown in Tables 1 and 2.

From the statistical results of Tables 1 and 2, the breast cancer classification prediction system based on ultrasonic image feature recognition constructed in this paper has certain effects. The system can be used for experimental diagnosis in the actual diagnosis of the hospital in the follow-up.

## 5. Conclusion

Medical image processing and analysis is a research hotspot in digital image processing and pattern recognition and an important application field of artificial intelligence and computer vision. The application of computer vision and machine learning in medical treatment can assist clinical diagnosis, reduce the contradiction between doctors and patients and the burden of doctors, improve the medical environment, and reduce treatment costs. Therefore, this research has very important application value. The clinical diagnosis of breast cancer is a complex, multivariate, and multifactorial process. There are many inspection items involved, and the physical and chemical indicators are complex. Therefore, it is necessary to consider the influence of multiple data sources and multiple factors. Moreover, we need to effectively integrate these data and dig out the potential information among different factors. These pieces of information complement each other to form a comprehensive and effective diagnosis basis. Finally, this paper constructs a breast cancer classification prediction model based on ultrasound feature recognition and combines experiments to verify the effectiveness of this diagnosis model.

## Figures and Tables

**Figure 1:** Coordinate system of the ultrasound probe system.

**Figure 2:** Schematic diagram before and after rendezvous and docking.

**Figure 3:** The coordinate system of rendezvous and docking with two ultrasonic probes.

**Figure 4:** The relationship diagram of the three coordinate systems.

**Figure 5:** Image coordinate system.

**Figure 6:** Schematic diagram of the small hole imaging model.

**Figure 7:** Breast cancer detection classification model based on ultrasonic image feature recognition.

**Figure 8:** Image analysis process diagram.

**Table 1:** The accuracy of breast cancer diagnosis based on ultrasonic image feature recognition.

Number	Diagnostic accuracy	Number	Diagnostic accuracy	Number	Diagnostic accuracy
1	93.9	26	92.0	51	96.1
2	97.9	27	90.7	52	95.9
3	96.1	28	96.1	53	96.2
4	94.0	29	89.9	54	95.7
5	94.5	30	91.6	55	95.9
6	89.9	31	93.6	56	94.3
7	96.9	32	89.9	57	97.5
8	93.4	33	90.8	58	94.7
9	97.5	34	94.9	59	94.4
10	94.7	35	91.1	60	93.2
11	94.5	36	94.9	61	94.8
12	97.2	37	94.4	62	90.4
13	89.0	38	96.5	63	89.2
14	89.9	39	89.4	64	94.5
15	93.0	40	94.4	65	91.1
16	94.0	41	89.0	66	92.9
17	93.8	42	90.4	67	96.1
18	92.5	43	95.4	68	90.5
19	95.6	44	94.1	69	90.2
20	90.6	45	93.4	70	92.2
21	91.3	46	90.0	71	89.8
22	94.5	47	94.4	72	94.6
23	89.2	48	97.2	73	92.1
24	95.7	49	94.7	74	90.6
25	94.7	50	95.4	75	93.0

**Table 2:** The accuracy of breast cancer classification based on ultrasonic image feature recognition.

Number	Classification accuracy	Number	Classification accuracy	Number	Classification accuracy
1	94.7	26	98.1	51	93.4
2	93.1	27	98.2	52	92.8
3	96.3	28	95.5	53	96.7
4	94.2	29	98.2	54	98.7
5	93.6	30	94.7	55	94.4
6	92.9	31	93.3	56	92.7
7	97.4	32	94.6	57	93.2
8	94.7	33	97.2	58	94.0
9	93.9	34	95.1	59	97.7
10	92.6	35	95.8	60	92.8
11	94.4	36	94.6	61	97.9
12	97.1	37	96.7	62	96.0
13	94.3	38	98.7	63	92.5
14	93.8	39	98.4	64	92.2
15	96.6	40	98.6	65	96.7
16	93.6	41	94.7	66	94.4
17	98.1	42	98.3	67	98.3
18	95.1	43	97.2	68	97.0
19	95.4	44	97.7	69	99.0
20	94.6	45	97.8	70	93.7
21	95.3	46	95.9	71	97.3
22	92.1	47	97.5	72	92.3
23	96.4	48	98.6	73	93.6
24	97.2	49	96.8	74	94.3
25	98.0	50	94.6	75	95.8

## Data Availability

The data used to support the findings of this study are included within the article.
